The article "Research on Kinetic Energy Recovery of Energy Vehicle ABS Solenoid Valve Based on the ELM Deep Learning Model" was retracted in 2023. Reasons: signs of a paper mill; suspected computer-generated content; unreliable results or conclusions; concerns about the data.

# Research on Kinetic Energy Recovery of Energy Vehicle ABS Solenoid Valve Based on the ELM Deep Learning Model

**DOI:** 10.1155/2022/6571085

**Published:** 2022-08-09

**Authors:** Chaoqun Tu, Lingli Zhang

**Affiliations:** Guangzhou Nanyang Polytechnic Vocational College, Guangzhou 510925, Guangdong, China

## Abstract

Aiming at the energy vehicle ABS kinetic energy recovery, this study optimizes the ABS system through the IPSO-ELM model, so that the energy vehicle can recover the energy generated by the ABS system to the greatest extent, so as to achieve the purpose of kinetic energy recovery and reduce energy consumption and vehicle cost. Based on the PSO-ELM model, a linear decreasing weighting method is introduced, and then, an IPSO-ELM model is proposed for the optimization analysis of ABS brake kinetic energy recovery. The results show that compared with the simple ELM model and PSO-ELM model, the simulation mean square error and relative error are significantly smaller, the generalization ability and prediction accuracy are higher, and the maximum relative error of the prediction result is 5.43% and the average relative error is 2.72%. The results confirm that the use of IPSO-ELM for ABS kinetic energy recovery optimization is extremely effective, and the study of ABS kinetic energy recovery for energy vehicles based on IPSO-ELM model optimization has strong application prospects and application potential.

## 1. Introduction

Although various countries are vigorously developing electric vehicles, the development momentum is still relatively slow. The main reason is that it is difficult to break through core technologies, such as solving energy problems. Energy source limitations increase the service life of the energy source and reduce the manufacturing cost of electric vehicles [1]. Under the current technical conditions, only the method of braking energy recovery can be used to increase the mileage of electric vehicles [2]. During the braking process, the ABS (Anti-lock Brake System) controls the brake pressure to keep the slip ratio near an optimal value when the wheels tend to lock, which can not only exert the maximum braking force but also ensure the handling and solidity of the vehicle [3]. When the energy vehicle is braked urgently, the wheel is subjected to the braking torque generated by the regenerative braking system and the braking torque generated by the friction brake at the same time [4]. How to distribute the relationship between friction braking and regenerative braking has become a key issue for regenerative braking systems [5]. If the braking energy regeneration system and the ABS system are reasonably coordinated and controlled, the economy of the vehicle can be improved, and driving safety can be enhanced [6]. Therefore, it is extremely necessary to study the kinetic energy recovery of ABS for electric new energy vehicles.

Unlike conventional vehicles, electric vehicle motor braking systems can provide regenerative braking force to recover energy. The goal of braking energy optimization is to recover as much energy as possible and improve vehicle economy on the premise of ensuring safe and stable braking of the vehicle. More energy can be recovered if more use of the motor is used for regenerative braking. Japan's research on in-wheel motor electric vehicles started relatively early. In the late 1990s, Japan's Toyota Motor Corporation began research on four-wheel in-wheel electric vehicles. In terms of control, by controlling the braking force of the four wheels, the ESC (Electronic Stability Control), the ASR (Anti-Slip Regulation), the ABS (Anti-lock Brake System), and related research studies on vehicle vertical vibration control [7, 8]. General Motors Corporation of the United States launched a hydrogen fuel cell four-wheel electric vehicle Sequel at the 2005 North American International Auto Show. Compared with traditional vehicles, the vehicle not only recovers vehicle solidity and traction presentation but also has a braking energy recovery function. Based on this idea, some scholars have designed a purely motor FE-RBS (Fully Electric Regenerative Braking System), which uses the motor as the only brake actuator [9]. However, because the regenerative braking system is limited by the external features of the motor and the state of responsibility of the battery, its braking torque working range is limited, and it may not be able to meet the driving braking requirements, and there are certain safety hazards, which limits the Wide application of FE-RBS. Therefore, most of the current braking energy recovery systems of electric vehicles are hydraulic and motor composite braking systems [10–12]. With the advancement of technology, ABS technology has been greatly improved, with higher control precision, stronger adaptability, smaller and smaller size, and lower and lower prices, ABS has become the standard of respective cars. Nowadays hybrid vehicles have begun to attract people's attention, and the world's major auto manufacturers have proposed regenerative braking and anti-lock braking strategies in the ABS technology of such vehicles, which not only improves the vehicle's performance. The dynamic performance can also be recovered as energy [13]. At the same time, with further research on the vehicle, the integration of ABS technology and driving anti-skid control device ASR has appeared, and ESP (Electronic Stability Control) has also been added to confirm the solidity of the vehicle on the basis of the application of ABS/ASR. With the development of technology, expanding the braking effect of the car, it is used together with the emerging EHB (Electronic Hydraulic Braking) and EMB (Electronic Mechanical Braking) to make the ABS respond faster [14]. At the same time, it is integrated with power electronic technology to better control the braking of the vehicle, such as adding EBD (brake force distribution device) to the ABS system, by calculating the adhesion on each wheel, effectively distributing the braking force of each wheel, thereby increasing the braking stability of the vehicle [15–17].

With the development of computer technology, ELM (Extreme Learning Machine) is widely used in various fields [18]. However, there are also some disadvantages. Randomly generating the weights and thresholds of hidden layer nodes may cause invalid hidden layer nodes, resulting in insufficient generalization ability [19, 20]. In order to search for higher precision and faster, this research proposes the adaptive weight method to improve the basic particle swarm algorithm, which effectively increases the diversity of particles and avoids falling into the local optimum. The IPSO was used to adjust the initial input weights and then establish the IPSO-ELM model, and apply the model to the research on kinetic energy recovery of the ABS solenoid valve of energy vehicles. The study has shown that the model has strong learning ability and high prediction accuracy. This method is very effective for optimizing the kinetic energy recovery of the ABS solenoid valve of energy vehicles.

## 2. Models and Methods

### 2.1. ELM Model

ELM is a machine learning method developed by Ding et al. [21] based on feedforward neural networks. The model contains input, hidden, and output layers. During the training process, it is no need to adjust the initial weights, only the need to set the number of nodes between the hidden layers, and the training can be completed by calculating the output weights by the least square method [22]. Related to the old-style neural network, this model has the rewards of faster training speed, higher accuracy, simpler parameter setting, and better generalization ability.

Assuming that there are *N* arbitrary samples (*X*_*i*_, *Y*_*i*_), among them, *X*_*i*_=$ ∈ $[*x*_*i*1_, *x*_*i*2_, *x*_*i*3_, ⋯,*x*_*in*_]^*T*^ ∈ *R*^*n*^, *Y*_*i*_=[*y*_*i*1_, *y*_*i*2_, *y*_*i*3_, ⋯,*y*_*in*_]^*T*^ ∈ *R*^*m*^_,_

(1) $$\begin{array}{c} \sum_{i=1}^{K}\beta_{i}g\left(W_{i}\times X_{i}+B_{i}\right)=t_{i}. \end{array}$$

Here, *K* is the number of nodes; *g*(*x*) is the activation function; *W*_*i*_=[*w*_*i*,1_, *w*_*i*,2_, *w*_*i*,3_, ⋯,*w*_*i*,*n*_]^*T*^ is the connection weight course between the input layer and the hidden layer; *β*_*i*_=[*β*_*i*,1_, *β*_*i*,2_, *β*_*i*,3_, ⋯,*β*_*i*,*n*_]^*T*^ is the joining mass vector among the output layer; *B*_*i*_ is the bias value of the *i*-th node in the neuron nodes. The approximate sample with zero error, which can be expressed as

(2) $$\begin{array}{c} \overset{N}{\underset{i=1}{\sum }}{\left\|t_{i}-Y\right\|}_{i}=0. \end{array}$$

That is, there are *β*_*i*_, *W*_*i*_, *B*_*i*_, so that the following formula holds.

(3) $$\begin{array}{c} \sum_{i=1}^{K}\beta_{i}g\left(W_{i}\times X_{i}+B_{i}\right)=Y_{i}. \end{array}$$

Equation (3) can be expressed as Equation (4) through a matrix.

(4) $$\begin{array}{c} H\beta =T. \end{array}$$

Here, *H* is the output matrix of the hidden layer; *β* is the output weight; *T* is the expected output. When the selected hidden layer excitation function *g*(*x*) in the model is infinitely differentiable, the input weights *ω* and hidden layer biases *B* can be randomly initialized, and the output weight *β* could be obtained by the minimum norm of the function as shown in the following formula:

(5) $$\begin{array}{c} \beta =H^{+}\times T. \end{array}$$

Here, *H*^+^ is the generalized inverse of Moore-Penrose of matrix *H*.

### 2.2. Improved Particle Swarm Optimization for Extreme Learning Machines (IPSO-ELM)

#### 2.2.1. Basic Particle Swarm Optimization (PSO)

The basic PSO procedure is resulting from the reproduction of simplified social models [23]. Pretentious that in the *d* dimensional pursuit planetary, there is a particle population of size *n*, and as (6) and (7), respectively [24].

(6) $$\begin{array}{c} V_{id}\left(t+1\right)=V_{id}\left(t\right)+c_{1}r_{1}\left(P_{id}\left(t\right)-X_{id}\left(t\right)\right)+c_{2}r_{2}\left(P_{gd}\left(t\right)-X_{id}\left(t\right)\right), \end{array}$$

(7) $$\begin{array}{c} X_{id}\left(t+1\right)=X_{id}\left(t\right)+V_{id}\left(t+1\right). \end{array}$$

In the formula, *t* is the number of iterations; *P*_i*d*_(*t*) is the different optimum explanation; *P*_*gd*_(*t*) is the global optimal solution; *c*_1_ and *c*_2_ are the knowledge issues; *r*_1_ and *r*_2_ are accidental figures consistently dispersed among [0,1].

#### 2.2.2. Improved Particle Swarm Optimization (IPSO)

Aiming at the phenomenon that the PSO algorithm is disposed too early adulthood, a linear decreasing weight method is proposed. Decreasing weight method, even if the apathy weight reductions linearly from small to large, its change formula is [25]

(8) $$\begin{array}{c} \omega =\omega_{\text{max}}-\frac{t\times \left(\omega_{\text{max}}-\omega_{\text{min}}\right)}{t_{\text{max}}}. \end{array}$$

Here, *ω*_max_ is the maximum apathy weight; *ω*_min_ is the minimum apathy weight; *t* is the existing repetition ladder. The calculation steps of the linear decreasing weight method are as follows.

(1) Arbitrarily generate the velocity and location of individual particles
(2) Assess the suitability value of individual particles, stock the place and appropriateness value of the particle in the individual dangerous value *P*_best_ of the element, and accept the separate location and suitability value of the optimal suitability value in all *P*_best_
(3) Update the velocity and position of the particle, and the control is exposed in the following equations.
  (9) $$\begin{array}{c} V_{i,j}\left(t+1\right)=\omega V_{i,j}\left(t\right)+c_{1}r_{1}\left(P_{i,j}\left(t\right)-X_{i,j}\left(t\right)\right)+c_{2}r_{2}\left(P_{g,j}\left(t\right)-X_{i,j}\left(t\right)\right), \end{array}$$
  (10) $$\begin{array}{c} X_{i,j}\left(t+1\right)=X_{i,j}\left(t\right)+V_{i,j}\left(t+1\right),j=1,2,\ldots ,n. \end{array}$$
(4) Update the weight, the calculation is shown in the following formula.
  (11) $$\begin{array}{c} \omega =\omega_{\text{max}}-\frac{t\times \left(\omega_{\text{max}}-\omega_{\text{min}}\right)}{t_{\text{max}}}. \end{array}$$
(5) When the model meets the disorder and reaches the rest, stop the search for corresponding consequence, else go back to step 3) to endure the study

#### 2.2.3. IPSO-ELM Model

The IPSO-ELM model aims to globally optimize the connection weights and hidden layer by relying on the advantages of the improved particle group procedure with strong worldwide exploration skill and fast junction speed [26] and then optimize the performance of the IPSO-ELM model. Prediction accuracy and prediction speed [27]. The specific operation steps are as follows, and the diagram of the IPSO-ELM model is revealed in Figure 1 [28].

1. Among the selected 35 groups of sample data
2. Initialize particle swarm parameters and generate particles randomly
3. Determine the ELM network and initialize the *w* and threshold of an extreme learning machine
4. Calculate the output weights to obtain the MSE
5. Take the MSE of the training output as the PSO fitness value
6. Initialize *P*_best_ and *g*_best_, update the speed and position of each particle according to *P*_best_ and *g*_best_, and calculate the fitness value corresponding to the current particle
7. Compare the current fitness value of the calculated particle swarm with the previously calculated *P*_best_ and *g*_best_, update the individual extremum and the global extremum, and finally get the position of the optimal particle
8. Assign the obtained optimal *w* and *b* to the extreme learning machine, predict, and output the test sample

### 2.3. Evaluation Standard

In this paper, NRMSE (Normalized Root Mean Square Error) [29] and NMAPE (Normalized Mean Absolute Percentage Error) [30] are used as prediction evaluation indicators. In addition, this study also used the mean squared error MSE to compare the three models. Its formula is as follows:

(12) $$\begin{array}{c} e_{t}=y_{t}-{\hat{y}}_{t},\\ \text{NMAPE}=\frac{1}{N}\sum_{t=1}^{N}\left|e_{t}\right|\times \frac{100}{C}\text{\%,}\\ \text{NRMSE}=\sqrt{\frac{1}{N}\sum_{t=1}^{N}e_{t}^{2}\times \frac{100}{C}\text{\%}}. \end{array}$$

Among them, *e*_*t*_ is the difference between the sample and the real value; *N* is the entire quantity of examples.

## 3. Test Analysis

The stability of ABS is affected by many factors, among which the main factors are the rotor speed *N*_ABS_ of the automobile anti-lock brake system, the speed of the automobile *V*_VEHICLE_, and the wheel radius *r*_wheel_, and the transmission ratio of the main reducer *i*_0_. These factors work together to affect the stability of ABS. and energy recovery performance, but there is a complex relationship between *N*_ABS_ and the transmission ratio of the final reducer, and it is difficult to make accurate judgments with traditional methods. The IPSO-ELM model could predict it, and four main influencing factors are made as the input restrictions model and output parameters model. 35 representative groups of sample data were selected, the first 30 groups were training data, and parameters were optimized, and the last 5 groups were test data. The detailed data are shown in Table 1.

To confirm the advantage of the IPSO-ELM, IPSO-ELM is associated with pure ELM and IPSO-ELM, as shown in Figure 2. It can be realized from Figure 2 that the IPSO-ELM has higher prediction accuracy. The predicted value of this model is nearby to the factual value, which is far better than ELM and IPSO-ELM. It can be realized from the comparison that the improved particle swarm algorithm is used to optimize the ELM model, which can advance the forecast accuracy of the ELM model and achieve a better prediction effect.

Based on MATLAB software, the MSE of each model can be obtained after running, and the MSEs of different models are compared, as exposed in Table 2. It can be realized from Table 2 that the MSE of the ELM model is 0.52376; the MSE of the PSO-ELM model is 0.45573; the MSE of the IPSO-ELM model is 0.09866. It can be realized that the IPSO-ELM model has high prediction accuracy, and has certain feasibility and effectiveness in the prediction of ABS stability and energy recovery performance.

Through MATLAB software, the iteration times of the IPSO-LEM model and PSO-ELM model are set to 100 times, and the error of each iteration is recorded and compared, as exposed in Figure 3. It can be gotten from Figure 3 that the iterative error of the IPSO-LEM model decreases successively. In the first 20 iterations, the error reduction range is large, and then the error reduction range is reduced, but it has been in a state of error reduction, and finally dropped to 0.043, indicating that the IPSO-LEM model has an ideal optimization effect. However, after 16 iterations of the PSO-LEM model, the iteration error does not change, and its value is stable at 0.13456, indicating that the forecast effect of the forecast model is not ideal and the prediction error is large.

The relation errors of the prediction results are compared in Table 3. The Error_max_ of the prediction results of the ELM model is 24.12%, and Error_average_ is 16.12%; the maximum relative error of the PSO-ELM model prediction results is 24.55%, and Error_average_ is 15.19%. Error_max_ of IPSO-ELM model prediction results is 5.43% and Error_average_ is 2.72%. It can be realized that the IPSO-ELM model has high prediction accuracy, the prediction results are relatively stable, the error among the forecasted actual is small, the model construction is reasonable, and the applicability is strong.

For the data of this study, comparing the ELM model and the classical method, it can be realized from the prediction consequences in Table 4 that when the prediction time is 24 h, the IPSO-ELM model has the highest accuracy. The NRMSE values decreased by 51.6% and 17.7%, respectively, and the NMAPE values decreased by 54.9% and 12.3%, respectively. When the prediction time was 48 h, the NRMSE values of the IPSO-ELM model decreased by 44.6% and 1.9%, and the NMAPE values decreased by 51.8% and 4.4%, respectively, compared with the PSO-ELM and ELM models. For the 72-hour power prediction, the NRMSE values of the IPSO-ELM model decreased by 31.6% and 7.1%, and the NMAPE values were reduced by 37.8% and 1.2%, respectively. For other classical models, the NRMSE and NMAPE values of the proposed model decreased the most within 24 h, followed by the second within 48 h.

## 4. Conclusion

Under the current technical conditions, only the method of braking energy recovery can be used to increase the mileage of electric vehicles. During the braking process, the ABS controls the brake pressure to keep the slip ratio near an optimal value when the wheels tend to lock, which can not only exert the maximum braking force but also ensure the handling and stability of the vehicle. If the braking energy regeneration system and the ABS system are reasonably coordinated and controlled, the economy of the vehicle can be improved, and the safety of driving can be enhanced. This study optimizes the ABS system through the IPSO-ELM model so that energy vehicles can maximize the energy generated by the ABS system, so as to achieve the purpose of kinetic energy recovery and reduce energy consumption and vehicle costs.

The conclusions are as follows. (1) On the basis of the PSO-ELM model, a linear decreasing weight method is introduced, and then, an IPSO-ELM model is proposed for the optimization analysis of ABS braking kinetic energy; (2) By comparing the prediction results of the three models with the actual values, the results show that compared with the pure ELM model and the PSO-ELM model, the IPSO-ELM model has significantly smaller simulation MSE and relative error and has higher generalization ability and prediction accuracy. The maximum relative error of IPSO-ELM model prediction results is 5.43%, and the average relative error is 2.72%. Compared with ELM and PSO-ELM, the error is lower. It is extremely effective to use IPSO-ELM for ABS kinetic energy recovery optimization.

## Figures and Tables

**Figure 1:** IPSO-ELM model diagram.

**Figure 2:** Comparison graph of predicted value and true value of different models.

**Figure 3:** Error change diagram of 100 iterations for different models.

**Table 1:** Training data and test data.

Serial number	*N*_ABS_	*V*_VEHICLE_	*r*_wheel_	*i*_0_	Serial number	*N*_ABS_	*V*_VEHICLE_	*r*_wheel_	*i*_0_
1	13.00	11.98	25	0.45	19	20.40	24.90	14	0.36
2	15.44	15.34	29	0.38	20	21.49	23.21	18	0.34
3	18.03	23.18	27	0.12	21	22.33	28.96	33	0.24
4	19.00	20.11	35	0.51	22	19.01	5.11	31	0.30
5	21.42	9.99	31	0.34	23	18.85	14.37	26	0.45
6	22.41	10.01	34	0.40	24	19.55	22.21	29	0.59
7	15.91	19.11	18	0.23	25	21.39	10.01	31	0.26
8	17.92	50.31	26	0.15	26	22.01	20.11	35	0.27
9	19.06	11.81	27	0.12	27	29.44	32.33	35	0.41
10	21.12	33.72	30	0.14	28	19.84	9.10	22	0.46
11	27.2	18.81	29	0.26	29	20.51	34.22	15	0.22
12	18.85	9.21	17	0.25	30	21.22	24.81	14	0.36
13	17.6	19.33	26	0.17	31	22.41	39.51	15	0.14
14	19.52	11.98	21	0.41	32	18.91	15.33	24	0.39
15	20.21	17.21	24	0.31	33	21.41	33.52	31	0.21
16	21.52	6.94	31	0.36	34	22.82	8.63	12	0.51
17	18.02	24.01	32	0.12	35	23.41	21.29	33	0.18
18	18.93	16.71	9	0.41					

**Table 2:** MSEs of different models.

Model	ELM	PSO-ELM	IPSO-ELM
MSE	0.52376	0.45573	0.09866

**Table 3:** Relative errors of prediction results of different models.

Sample number	Actual value	ELM	PSO-ELM	IPSO-ELM	Relative error (ELM and true value) (%)	Relative error (PSO-ELM and true value) (%)	Relative error (IPSO-ELM and true value) (%)
1	1.560	1.484	1.361	1.596	4.9	12.74	2.32
2	1.630	1.239	1.341	1.615	24.12	17.67	0.91
3	1.280	1.491	1.447	1.277	16.51	13.07	0.27
4	1.030	1.261	1.283	1.086	22.36	24.55	5.43
5	1.250	1.413	1.350	1.192	13.06	8.02	4.66
Average value	1.350	1.377	1.357	1.353	16.12	15.19	2.72

**Table 4:** Experiment results with other models.

Evaluation criteria	Model	Prediction duration (h)		
		24	48	72
NRMSE	ELM	48.56	56.72	46.43
	PSO-ELM	28.53	32.02	34.17
	IPSO-ELM	23.47	31.39	31.73

NMAPE	ELM	41.33	50.65	39.71
	PSO-ELM	21.23	25.52	24.99
	IPSO-ELM	18.60	24.39	24.68

## Data Availability

The data used to support the findings of this study are available from the corresponding author upon request.
